The article "The Awareness of the Human Papillomavirus Infection and Oropharyngeal Cancer in People to Improve the Health Care System at Al Qunfudhah Region, Kingdom of Saudi Arabia" was retracted in 2023. Reasons: signs of a paper mill; compromised peer review; unreliable results or conclusions.

# The Awareness of the Human Papillomavirus Infection and Oropharyngeal Cancer in People to Improve the Health Care System at Al Qunfudhah Region, Kingdom of Saudi Arabia

**DOI:** 10.1155/2021/5185075

**Published:** 2021-10-19

**Authors:** Ali Maeed Alshehri, Muaddiyah Mohammed Ahmed Alamri, Amal Ahmed Mahdi Alharazi, Adnan Mohammed Essa Alhazmi, Reem Mohammed Hassan Alfaqih, Abdulrahim Ali Ibrahim Alzaylaee, Salihah Harb Awadh Almarhabi, Hassan Mohammed Hassan Alfaqih, Amaal Ali Khneen Alderhami, Mariam Harb Awadh Almarhabi, Abdullah Alsllami

**Affiliations:** ^1^Otolaryngology College of Medicine, King Khalid University, Abha, Saudi Arabia; ^2^Qunfudah Medical College, Al Qunfudhah, Saudi Arabia; ^3^Ministry of Health, Al Qunfudhah, Saudi Arabia

## Abstract

With 14 million new infections each year, the human papillomavirus (HPV) is the most common sexually transmitted infection (STI) among both men and women in the United States (US). Infections with the human papillomavirus (HPV) are responsible for a considerable portion of the global cancer burden. HPV-related oral malignancies are on the rise around the world, according to epidemiological studies. To provide accurate advice to their patients, dental practitioners require thorough, up-to-date HPV-related knowledge. *Methods.* In this cross-sectional study, data were collected by the purposely constructed questionnaire. A questionnaire composed of the demographic items and items related to the awareness and knowledge about Human papillomavirus. The questionnaire was constructed after a series of discussions between the panel of experts. This panel was composed of a subject specialist, researcher, and language expert. The Cronbach alpha of the questionnaire was calculated. The study will be conducted in the Al Qunfudhah. *Results.* The Cronbach alpha of the questionnaire was 0.72. Out of a total of 550 respondents, with a mean (SD) age of 47.5 (11.5), the female respondents were 167 (30.4%) while male were 383 (69.6%). 20.5% of the respondents (out of 550) were having awareness of HPV. *Implications.* Knowledge of HPV-related oral cancer is critical, and it is advised to be taught as part of dental students' basic curriculum and clinical training. This problem can be solved by better educational training programs. Knowledge of HPV-related oral cancer is critical, and it is advised to be taught as part of dental students' basic curriculum and clinical training.

## 1. Introduction

With 14 million new infections each year, the human papillomavirus (HPV) is the most common sexually transmitted infection (STI) among both men and women in the United States (US). Infections with the human papillomavirus (HPV) are responsible for a considerable portion of the global cancer burden. HPV-related oral malignancies are on the rise around the world, according to epidemiological studies. To provide accurate advice to their patients, dental practitioners require thorough, up-to-date HPV-related knowledge.

The article "The Awareness of the Human Papillomavirus Infection and Oropharyngeal Cancer in People to Improve the Health Care System at Al Qunfudhah Region, Kingdom of Saudi Arabia" was retracted in 2023. Reasons: signs of a paper mill; compromised peer review; unreliable results or conclusions.

TSeropositive men are more likely to acquire penile and anal cancer after contracting HPV, and other studies found that HIV–HPV seropositive people are 60 percent more likely to get cancer than healthy people. 10 heterosexual HPV-positive persons, on the other hand, can transfer the virus to their female partners, which is linked to cervical cancer in these women. Skin-to-skin or skin-to-mucosa contact is the most common way for HPV infections to spread. More than 200 HPV kinds have been identified thus far [1].

The epidemiology of HPV in Saudi Arabian women is poorly understood, and there are few publications in this community about HPV prevalence, detection, and genotyping, as well as attitudes about screening.

In 2018, a study in Saudi Arabia discovered that oropharyngeal cancer is more common in men than in women. According to the findings, there were 12 new cancer cases each year in men, with a crude incidence rate of 0.1, an age-standardized incidence rate of 0.1, and cumulative risk (%) of 0 at 75 years old. The annual number of new cancer cases in females was 6, with a crude incidence rate of 6 and an age-standardized incidence rate of 0 percent [2].

Based on their carcinogenic potential, HPVs are categorized into two categories: high risk and low risk. High-risk strains include HPV 16, 18, 31, 33, 35, 39, 45, 51, 52, 56, 58, 59, 68, 73, and 82 [3]. HPV 6 and HPV 11 are low-risk HPV strains that produce genital and respiratory tract warts as well as modest cervical abnormalities [4–6]. More than 90% of HPV-related malignancies are caused by HPV strains 16 and 18 [7].

Oncogenic strains of the HPV are associated with at least six different cancers including oropharyngeal, anal, cervical, vaginal, vulvar, and penile cancers [7–9]. The landscape of head and neck squamous cell carcinoma is changing, with the human papillomavirus (HPV) being a more common cause of oropharyngeal carcinoma [10]. Oropharyngeal cancer caused by HPV accounts for around 4.5% of all cancers worldwide, with an estimated 630,000 new cases diagnosed per year [11]. Human papillomavirus (HPV) is implicated in up to 25% of HNCs, with HPV accounting for up to 60% of cases in oropharyngeal carcinoma (OPC) [12]. Approximately, 75% of HPV-associated oropharyngeal cancer patients are male [8].

HPV has been discovered as an oncogenic driver in HNC, according to a study conducted in Canada in 2016, and the prevalence of HPV + HNC, particularly HPV + OPC, is growing [12]. In 2005, Candotto published a systematic review analysis that showed HPV DNA in 35.6 percent of oropharyngeal malignancies, with HPV type 16 accounting for the great majority of HPV-positive cases (87 percent) [13]. Oral sexual contact and open-mouth kissing are key risk factors for oral HPV infection and HPV-OPC, according to a study done in the United States in 2017 [10]. Few studies looked at the sociodemographic traits or sexual habits of Saudi women who have HPV, according to a study conducted in Riyadh, Saudi Arabia, in 2016. The researchers revealed a significant frequency of HPV infection, with key risk factors including smoking and having many relationships [14]. By 2020, the incidence of HPV-positive OPSCC will outnumber cervical cancer, and by 2030, HPV will be linked to 50% of all head and neck cancers, according to Chaturvedi et al. [15].

The article "The Awareness of the Human Papillomavirus Infection and Oropharyngeal Cancer in People to Improve the Health Care System at Al Qunfudhah Region, Kingdom of Saudi Arabia" was retracted in 2023. Reasons: signs of a paper mill; compromised peer review; unreliable results or conclusions.

Fortunately, three HPV vaccinations have been developed to protect against up to nine different strains of HPV [1]. The quadrivalent vaccine prevents around 70% of cervical cancer, whereas the 9-valent vaccine prevents about 80% of cervical cancer, 66 percent of oropharyngeal cancer, 88 percent of anal cancer, and 57% of penile cancer [8]. Even though HPV vaccinations have been available for women since 2006 and males since 2011, vaccine uptake remains low [7].

Because of a lack of proper awareness and understanding regarding HPV-related infections and malignancies, we need to enhance the knowledge According to recent studies conducted in Florida and Italy. Very few respondents were aware of the presence and availability of an HPV vaccine [15, 16]. Only 21.5 percent of patients attending primary care clinics in Saudi Arabia were aware that there is an HPV vaccine [17]. Multiple studies discovered a link between gender, younger age, and higher levels of education and awareness of HPV disease and immunizations [7–9, 11, 18, 19]. According to a study conducted in the United States, only 29.9% of people were aware that HPV increases the risk of head and neck malignancies, while 42.4 percent mistook HPV for HIV, and only 25.1 percent received HPV knowledge from a health care provider [19].

In a similar study conducted on physicians in Saudi Arabia in 2017–2018, it was discovered that physicians are only partially aware of the evident dangers of HPV infection to the Saudi population. Physicians, on the other hand, frequently reported modest levels of concern about HPV infection. Lack of information about the vaccine and concerns about vaccine safety and cost were cited as reasons for rejecting the vaccine, demonstrating a widespread unfavorable attitude about the HPV vaccine that may underplay clinicians' role in prescribing immunization for their patients [20].

The article "The Awareness of the Human Papillomavirus Infection and Oropharyngeal Cancer in People to Improve the Health Care System at Al Qunfudhah Region, Kingdom of Saudi Arabia" was retracted in 2023. Reasons: signs of a paper mill; compromised peer review; unreliable results or conclusions.

Due to the paucity of information available on the extent of people's awareness and knowledge of HPV disease and vaccines in Al Qunfudhah and the lack of published research on this point, in this study, we aim to assess the extent of people's awareness and knowledge of the HPV diseases, methods of transmission, vaccines, and related cancers.

### 1.1. Main Objectives

1. To assess the awareness of HPV infection and oropharyngeal cancer in people in the Al Qunfudhah region, Kingdom of Saudi Arabia.
2. To estimate the knowledge and attitude of HPV infections, related cancer, and vaccination in people in the Al Qunfudhah region, Kingdom of Saudi Arabia.
3. To calculate the prevalence of HPV infection in people in the Al Qunfudhah region, Kingdom of Saudi Arabia.
4. To assess the effect of education on the participant's knowledge and awareness about HPV infections.

## 2. Methods

In this cross-sectional study, data were collected by the purposely constructed questionnaire, a questionnaire composed of the demographic items and items related to the awareness and knowledge about the Human papillomavirus. A questionnaire was constructed after a series of discussions between the panel of experts. This panel was composed of a subject specialist, researcher, and language expert. Cronbach alpha of the questionnaire was calculated. The study was conducted in the Al Qunfudhah region of Saudi Arabia. The questionnaire included items related to the awareness of HPV, demographic variables, the vaccine, and other items.

After the collection of data, data were coded and entered in the SPSS ver. 20 software for descriptive statistics (mean standard deviation, frequencies, and %s were computed), to measure the significance differences *t*-test and chi-square test was used at 5% level of significance. Data were collected from the patients who visit the Primary Health Care Center at Al Qunfidah city of Saudi Arabia and from the general public of A Qunfidah city of Saudi Arabia through an electronic version of the questionnaire. Ethical approval was obtained from King Khalid University, Saudi Arabia. The study duration was from January 2021 to April 2021.

## 3. Results

The Cronbach alpha of the questionnaire was 0.72. Out of a total of 550 respondents, with mean (SD) age of 47.5 (11.5), the female respondents were 167 (30.4%) while males were 383 (69.6%). We observed that 20.5% (out of 550) respondents were having awareness of HPV. We observed a significant difference while comparing gender with awareness questions. Further, 29% (out of 113 respondents) agreed that HPV vaccination can prevent oropharyngeal cancer.

The article "The Awareness of the Human Papillomavirus Infection and Oropharyngeal Cancer in People to Improve the Health Care System at Al Qunfudhah Region, Kingdom of Saudi Arabia" was retracted in 2023. Reasons: signs of a paper mill; compromised peer review; unreliable results or conclusions.

Figure 1 20.5% of respondents (out of 550) were having awareness of HPV.

In Table 1, we compared the demographic variables with the awareness regarding HPV and oropharyngeal cancer, we have observed the significant difference in gender and age variable regarding the HPV and, similarly, we observed significant differences while comparing awareness level of oropharyngeal cancer with age, while other variables are insignificant.

Figure 2 shows that 30% opted that they will likely receive vaccination against HPV, 25% opted somewhat, 19% opted very likely, 8% opted unlikely, 9% opted very unlikely, and 10% opted somewhat unlikely.

Table 2 depicts that 11%, 20%, 16%, 16%, 25%, 11%, and 10% have a perception that HPV can cause anal, cervical, prostate, vaginal, breast, laryngeal, lung, and skin cancers, respectively.

Out of 113 respondents (those who were aware of HPV) opted that HPV can cause HIV aids (24% agreed), 49% had no idea, and 27% disagree (Figure 3).

Figure 4 depicts that 29% (out of 113 respondents) agreed that HPV vaccination can prevent oropharyngeal cancer.

Figure 5 shows that only 2% (out of 550) had suffered from HPV.

Figure 6 shows that 23% (out of 113) admitted that HPV always has clear signs and symptoms.

## 4. Discussion

In this study, our major aim was to assess the awareness and attitude towards HPV infections, diseases, and vaccination associated with HPV. In the United States, roughly, 42% of persons aged 18 to 59 have genital human papillomavirus (HPV) infections, while about 7% have oral HPV infections [21, 22]. According to experts, 80 percent of sexually active persons are infected with HIV. Every year, 14 million new HPV infections are diagnosed. In Saudi Arabia, one study stated that the human papillomavirus (HPV) was identified in 43% of the samples, which is in contrast to the findings of our study in our study indicating that only 2% of the respondents had suffered from HPV infections [23–25].

HPV is a group of DNA viruses that infect basal epithelial cells and cause benign and malignant diseases of the skin, anogenital mucosae, and upper aerodigestive tract mucosae. 4–6 HPV types 16, 18, 31, 33, 35, 39, 45, 51, 52, 56, 58, and 59 have been classified as carcinogenic, while HPV68 has been classified as possibly carcinogenic, based on epidemiological research and mechanistic evidence. HPV is the cause of nearly all cervical cancers, as well as a significant number of other anogenital and oropharyngeal malignancies. Understanding the cancer burden caused by HPV can help to improve HPV vaccine and HPV-based cervical screening programs. In our study, we found that a reasonable quantity of the respondents agreed that HPV can cause different types of cancers [25–28].

The article "The Awareness of the Human Papillomavirus Infection and Oropharyngeal Cancer in People to Improve the Health Care System at Al Qunfudhah Region, Kingdom of Saudi Arabia" was retracted in 2023. Reasons: signs of a paper mill; compromised peer review; unreliable results or conclusions.

On the role of HPV in cervical cancer, there is significant epidemiological evidence (Munoz, 2000). In our study, a significant number of the respondents agreed to have a vaccination for HPV as the study stated that. Vaccine efficacy against high-risk HPV types (HPV) has been found to range from 90 to 99 percent in preventing cervical cancer in numerous clinical trials and systematic reviews around the world (CIN). These assessments also provide ample evidence of the vaccinations' safety [29].

Many underdeveloped nations have a low uptake of HPV vaccination due to factors such as a decreased perceived risk of cervical cancer, a lack of vaccine availability, and exorbitant costs. However, one of the most critical deciding reasons for low vaccination uptake is a lack of proper knowledge regarding the role of HPV in the development of cervical carcinoma and the HPV vaccine [30, 31].

According to numerous studies conducted among physicians and nurses, the most crucial aspects evaluated by clinicians when considering the HPV vaccine were effectiveness and side effects/safety. Government recommendations and expenses were also taken into account. The importance of clear government advice and cost were also examined. Many of these studies underlined the need for additional information regarding the virus, cervical cancer, and vaccination to boost people's readiness to suggest it [32–35].

The signs and symptoms of HPV are usually not visible, which is also stated in our study that the majority of the respondents were unfamiliar regarding the signs and symptoms of HPV [36].

In our study, a reasonable volume of the respondents agreed that the HPV vaccination is a method for preventing oropharyngeal cancer which is also proof by the study stating that HPV VLP vaccinations of the current generation (HPV 16/18) have the potential to prevent >90% of HPV-positive oropharyngeal malignancies. Men and possibly women should be included in clinical trials evaluating the efficacy of HPV VLP vaccinations for the prevention of incident and chronic oral HPV 16 infection [37].

In women who live in a place where both illnesses are common, cervical HPV infection is linked to HIV infection. Much research is needed to determine whether the reported link is causative. In our study, 24% of the population agreed that cervical HPV infection is linked to HIV infection.

Education might play an important role in having HPV vaccination and avoiding cancers; in our study, university graduates having more desire to get vaccinations of HPV which is inconsistent with the findings of the study stating that to achieve immunization, educational programs aimed at health care practitioners, as well as cost-cutting initiatives and clear government rules, are urgently required [38].

The article "The Awareness of the Human Papillomavirus Infection and Oropharyngeal Cancer in People to Improve the Health Care System at Al Qunfudhah Region, Kingdom of Saudi Arabia" was retracted in 2023. Reasons: signs of a paper mill; compromised peer review; unreliable results or conclusions.

## 5. Conclusion

These findings imply that respondents have significant HPV-related knowledge gaps, which limit their ability to intervene in oropharyngeal primary prevention initiatives. The findings of this study recommend that HPV-related instructional content be included and standardized in school, college, and university curricula. This problem can be solved by better educational training programs. Knowledge of HPV-related oral cancer is critical, and it is advised that it should be taught as part of dental students' basic curriculum and clinical training. This research will serve as a foundation for future research and therapies. Medical students should do a follow-up comparative study.

## Figures and Tables

**Figure 1:** Do you have some awareness regrading HPV?

**Figure 2:** Vaccination against HPV is now available. How likely is it to receive the vaccine in the future?

**Figure 3:** HPV and HIV.

**Figure 4:** The HPV vaccination is a method for preventing oropharyngeal cancer.

**Figure 5:** Have you ever had HPV?

**Figure 6:** HPV always has clear signs and symptoms.

**Table 1:** Demographic variables.

Variables		Do you have some awareness of HPV?			Have you ever heard of oropharyngeal cancer?		
		Yes	No	*p* value	Yes	No	*p* value
Age	18–24 years old	22	36	0.017	38	20	0.019
	25–40 years old	44	206		188	62	
	Over 40 years old	47	195		206	36	

Gender	Female	48	119	0.004	124	43	0.301
	Male	65	318		308	75	

Education	Primary level	0	7	0.316	0	7	0.449
	Middle school	6	11		14	3	
	High school	18	100		89	29	
	University level	89	319		329	79	

Monthly income	10,000–14,999	35	136	0.171	131	40	0.002
	15,000–19,999	17	77		80	14	
	20,000 or more	21	51		68	4	
	5000–9999	10	65		51	24	
	Less than 5000	30	108		102	36	

Marital status	Married	84	358	0.14	357	85	0.137
	Single	26	64		64	26	
	Widow	3	15		11	7	

**Table 2:** HPV and cancers.

		Frequency	%
HPV can cause anal cancer	False	26	5
	I do not know	461	84
	True	63	11

HPV can cause cervical cancer	False	21	4
	I do not know	421	77
	True	108	20

HPV can cause prostate cancer	False	36	7
	I do not know	452	82
	True	62	11

HPV can cause vaginal cancer	False	22	4
	I do not know	434	79
	True	94	16

HPV can cause breast cancer	False	36	6
	I do not know	428	78
	True	86	16

HPV can cause laryngeal cancer	False	19	3
	I do not know	392	71
	True	139	25

HPV can cause lung cancer	False	41	7
	I do not know	451	82
	True	58	11

HPV can cause skin cancer	False	40	7
	I do not know	453	82
	True	57	10

The article "The Awareness of the Human Papillomavirus Infection and Oropharyngeal Cancer in People to Improve the Health Care System at Al Qunfudhah Region, Kingdom of Saudi Arabia" was retracted in 2023. Reasons: signs of a paper mill; compromised peer review; unreliable results or conclusions.

## Data Availability

The data will be available upon reasonable request.
